The article "Deep Unsupervised Hashing for Large-Scale Cross-Modal Retrieval Using Knowledge Distillation Model" was retracted in 2023. Reasons: signs of a paper mill; compromised peer review; unreliable results or conclusions.

# Deep Unsupervised Hashing for Large-Scale Cross-Modal Retrieval Using Knowledge Distillation Model

**DOI:** 10.1155/2021/5107034

**Published:** 2021-07-17

**Authors:** Mingyong Li, Qiqi Li, Lirong Tang, Shuang Peng, Yan Ma, Degang Yang

**Affiliations:** College of Computer and Information Science, Chongqing Normal University, Chongqing 401331, China

## Abstract

Cross-modal hashing encodes heterogeneous multimedia data into compact binary code to achieve fast and flexible retrieval across different modalities. Due to its low storage cost and high retrieval efficiency, it has received widespread attention. Supervised deep hashing significantly improves search performance and usually yields more accurate results, but requires a lot of manual annotation of the data. In contrast, unsupervised deep hashing is difficult to achieve satisfactory performance due to the lack of reliable supervisory information. To solve this problem, inspired by knowledge distillation, we propose a novel unsupervised knowledge distillation cross-modal hashing method based on semantic alignment (SAKDH), which can reconstruct the similarity matrix using the hidden correlation information of the pretrained unsupervised teacher model, and the reconstructed similarity matrix can be used to guide the supervised student model. Specifically, firstly, the teacher model adopted an unsupervised semantic alignment hashing method, which can construct a modal fusion similarity matrix. Secondly, under the supervision of teacher model distillation information, the student model can generate more discriminative hash codes. Experimental results on two extensive benchmark datasets (MIRFLICKR-25K and NUS-WIDE) show that compared to several representative unsupervised cross-modal hashing methods, the mean average precision (MAP) of our proposed method has achieved a significant improvement. It fully reflects its effectiveness in large-scale cross-modal data retrieval.

## 1. Introduction

At present, the mobile Internet and social networks are developing rapidly, and smart terminals, video surveillance, etc., are widely used, so massive multimedia data (images, texts, videos, audios, etc.) are generated every day. Therefore, cross-modal retrieval [1–5] has received extensive attention and applications. The goal of cross-modal retrieval is to search for semantically related instances from different modalities, for example, using text instances as query points to find images with the same semantics. In order to meet the retrieval requirements of fast retrieval speed and small storage space in the real world, the hashing method uses binary hash code to represent the original data, and the time complexity can reach constant or sublinear in the application of approximate nearest neighbor search. It is widely used for cross-modal retrieval.

The article "Deep Unsupervised Hashing for Large-Scale Cross-Modal Retrieval Using Knowledge Distillation Model" was retracted in 2023. Reasons: signs of a paper mill; compromised peer review; unreliable results or conclusions.

Cross-modal hashing [1, 5–8] is one of the most popular retrieval methods, which maps large-scale high-dimensional cross-modal data to a common binary hash space. By compressing each instance into a short binary code, the cross-modal hash method greatly improves retrieval speed and storage efficiency. According to whether to use supervised information, cross-modal hashing can be divided into two methods: unsupervised and supervised methods. Supervised methods' [3, 6, 9] manual labeling requires expensive labor costs and calculations, and semantic labels can be further used to learn more consistent hash codes for semantically related cross-modal data, which usually produces more accurate results. The unsupervised method [7, 10, 11] greatly reduces the computational cost and is easier to deploy to actual scenarios, while achieves lower performance.

In recent years, due to the excellent performance of deep neural network in many classical scenarios [12, 13], it can be used as a nonlinear hash function to realize end-to-end feature representation and hashing coding, so deep cross-modal hashing has attracted more and more attention and gained great development. Compared with the shallow method using manually extracted features to learn the hash code, the deep cross-modal hash method [2, 5, 14, 15] directly learns the mapping function from the original data to the hamming space, which is more effective in finding the potential relationship between the original data and the hashing code.

Although unsupervised cross-modal hashing has advantages in reducing the burden of manual annotation of data and is more widely used in real-world scenarios, its accuracy is often less than satisfactory, especially when compared with supervised methods. The main reason is the lack of pairwise similarity knowledge of training data pairs. The output of unsupervised models usually contains some inaccurate semantic information. Therefore, we focus on improving the accuracy of unsupervised learning methods, which have a wider range of applications in the real world.

In this paper, we propose a novel unsupervised cross-modal hashing method based on semantic alignment using knowledge distillation (SAKDH), which solves the problem of lack of supervised information by distilling data pairs with reliable semantic similarity. Specifically, our approach consists of two modules: the teacher module is an unsupervised module, and the student module is a supervised module; the teacher module gets the distillation data, which is then used to supervise the training of the student module.

The article "Deep Unsupervised Hashing for Large-Scale Cross-Modal Retrieval Using Knowledge Distillation Model" was retracted in 2023. Reasons: signs of a paper mill; compromised peer review; unreliable results or conclusions.

Drawing on the idea of knowledge distillation, we use the teacher and student model to combine the advantages of both approaches (supervised and unsupervised). In the supervised methods, the most important information is the similarity between each pair of cross-modal data. After training, the unsupervised teacher model can output the feature vectors of each instance, and the similar information can be obtained by calculating the distance between their feature vectors. In short, the main contributions of this paper are as follows:

1. We migrated knowledge distillation into the CMH scenario and proposed a novel unsupervised deep cross-modal hashing approach, which can reconstruct the similarity matrix using the hidden correlation information of the pretrained unsupervised teacher model, and the reconstructed similarity matrix can be used to guide the supervised student model. This is a novel method of using unsupervised methods to guide supervised CMH.
2. An unsupervised semantic alignment hashing method is adopted for the teacher model, which can enhance the discrimination ability of the hash code. The student model adopts the joint loss of pairwise and triplet; these loss functions apply not only to intermodal, but also to intramodal. This can make the original semantically related instances, and its hash code also retains the semantic relevance well.
3. Experimental results on two extensive benchmark datasets (MIRFLICKR-25K and NUS-WIDE) show that compared to several representative unsupervised cross-modal hashing methods, the Mean Average Precision (MAP) of our proposed method has achieved a significant improvement. It fully reflects its effectiveness in large-scale cross-modal data retrieval.

## 2. Related Work

Cross-modal retrieval methods can be divided into two categories: unsupervised methods and supervised methods. Supervised CMH methods [9, 16–20] generally use the label information of the input image-text pair to maximize their semantic similarities in the hamming space and use some methods to make the difference modalities learn a unified hash code, which is effective in cross-modal retrieval, and has been extensively studied. Because of the excellent performance of deep neural networks in nonlinear representation learning, many supervised deep cross-modal hashing methods [15, 21] have achieved excellent performance in cross-modal retrieval tasks. These supervised methods can obtain relevant information from semantic labels of images and text, thus achieving better performance. However, obtaining large numbers of such labels is often expensive and tricky, making the supervised approach impractical in real-world applications. Compared with the supervised method, the unsupervised cross-modal methods [10, 22, 23] does not rely on semantic tags during the training process, making it easier to deploy to actual scenarios. However, it is more difficult to learn, and related research is relatively insufficient.

The article "Deep Unsupervised Hashing for Large-Scale Cross-Modal Retrieval Using Knowledge Distillation Model" was retracted in 2023. Reasons: signs of a paper mill; compromised peer review; unreliable results or conclusions.

### 2.1. Unsupervised Shallow Cross-Modal Hashing

Unsupervised cross-modal hashing methods can be divided into shallow methods and deep methods. CVH [7] is a representative of the early shallow unsupervised methods, using cross-view hashing to learn shallow hash functions. IMH [11] uses spectral hashing to transform heterogeneous cross-modal data into hamming space for unified learning. CMFH [24] learns a unified hash code by collaboratively decomposing the feature matrix of cross-modal data. CCQ [25] jointly finds the correlation maximum mapping that transforms different modalities into isomorphic potential spaces and learns the compound quantizer that transforms isomorphic potential features into compact binary codes. LSSH [26] uses sparse coding to capture the salient structure of the image and obtains the underlying concepts of the text through matrix decomposition, exploring the semantic information hidden in the data. These methods cannot effectively capture the complex nonlinear mapping of different modal data to the hamming space, so many unsupervised cross-modal methods introduce deep neural networks into the learning of hash codes to construct a nonlinear mapping from data to hash codes.

### 2.2. Unsupervised Deep Cross-Modal Hashing

With the development of deep learning, deep cross-modal hashing methods have become mainstream in recent years [10, 22, 23, 27–30]. DBRC [31] proposes deep binary reconstruction cross-modal hashing to maintain consistency within and between modalities. UDCMH [28] jointly optimizes the feature learning and binarization process and learns a unified binary code. DJSRH [29] constructs a joint semantic similarity matrix based on the neighborhood information of different modalities and proposes deep joint semantic reconstruction hashing for cross-modal retrieval. JDSH [27] fully preserves the cross-modal semantic association between instances by constructing the joint-modal similarity matrix and similarity decision and weighted method based on distribution. UKD [30] uses output generated by unsupervised methods to guide supervisory methods and make use of teacher-student optimization for propagating knowledge. UGACH [22] and UCH [32] train the networks in an adversarial learning manner, through the way of cross-modal adversary. MGAH [33] extends UGACH to multimodal retrieval among five modalities, but these adversarial methods have problems such as difficulty in training and high time complexity.

The article "Deep Unsupervised Hashing for Large-Scale Cross-Modal Retrieval Using Knowledge Distillation Model" was retracted in 2023. Reasons: signs of a paper mill; compromised peer review; unreliable results or conclusions.

Although unsupervised cross-modal hashing has advantages in reducing the burden of manual annotation of data and is more widely used in real-world scenarios, its accuracy is often less than satisfactory, especially when compared with supervised methods. The main reason is the lack of pairwise similarity knowledge of training data pairs. The output of unsupervised models usually contains some inaccurate semantic information. Therefore, we focus on improving the accuracy of unsupervised learning methods, which have wider applications in real-world scenarios. Inspired by the idea of knowledge distillation, we use the output of the unsupervised model to guide the supervised model. That is, we use distilled knowledge to aid model training.

## 3. Proposed Method

Knowledge distillation can use a more complex model (teacher) that has been trained to guide a lighter model (student) training, so as to reduce the size of the model and computational resources, while trying to maintain the accuracy of the original large model. Our proposed SAKDH method, summarized in one sentence, is to train a student network with the soft label output of teacher network. In this work, we use the output of the unsupervised method to guide the supervised cross-modal hashing method.  Figure 1 shows the proposed SAKDH framework.

### 3.1. Soft Similarity

The key to CMH is to identify which image/text pairs are semantically relevant and which are semantically unrelated, enabling the model to learn to pull the features of the correlation pair closer together in the common space. A common method is to define a similarity matrix *S* ∈ {0,1}^*n*×*n*^, *s*_*ij*_=1 indicates that these image/text pairs are positive sample pairs and vice versa. This way is called hard similarity. If *S* ∈ [0,1]^*n*×*n*^, *s*_*ij*_ is a real value between [0, 1]; this is what we call soft similarity. In our distillation model, the output is soft similarity. We can use the example in Figure 2 to understand the idea of soft similarity and hard similarity. In addition to positive tag, negative tags also carry a lot of information; for example, the corresponding probability of some negative tags is far greater than that of others. In the traditional training process (hard similarity), all negative tags are 0. In other words, the training way of SAKDH makes each sample bring more information to the student network than the traditional training method.

### 3.2. Problem Definition

Let us start with some of the notations used in this paper. Assume that we have *n* instances which can be denoted as *O*={*o*_*i*_}_*i*=1_^*n*^, and each instance can be described by an image-text pair *o*_*i*_ ∈ (*v*_*i*_, *t*_*i*_). We use *F*^*∗*^={*f*_*i*_^*∗*^}_*i*=1_^*n*^ ∈ *ℝ*^*n*×*D*^*∗*^^, *∗* ∈ {*v*, *t*}, to represent the feature vectors extracted from the ImageNet_T or TextNet_T, where *D*^*∗*^, *∗* ∈ {*v*, *t*}, denotes the dimension of image or text modality feature space. In addition, *B*^*∗*^={*b*_*i*_^*∗*^}_*i*=1_^*n*^ ∈ {−1,1}^*n*×*c*^, *∗* ∈ {*v*, *t*}, denotes the hash codes generated of image or text modality, where *c* denotes code length.

The article "Deep Unsupervised Hashing for Large-Scale Cross-Modal Retrieval Using Knowledge Distillation Model" was retracted in 2023. Reasons: signs of a paper mill; compromised peer review; unreliable results or conclusions.

### 3.3. Unsupervised Knowledge Distillation

In the unsupervised teacher model, we shared the idea of DSAH [34]. In order to make full use of image-text pairs, we designed an unsupervised deep semantic alignment loss function, including similar semantic alignment loss and diagonal semantic alignment loss. It is possible to align the similarity between the features with the similarity between the hash codes at the same time.

In unsupervised cross-modal hashing methods, the instance's annotation is not available. The features extracted from the deep neural network contain rich semantic information, so we can construct the similarity matrix by using the features without annotation. In this paper, to describe the neighbor relations in the hamming space, we calculate the pairwise cosine similarity matrices and define *S*_*v*,*v*_^*B*^ for the image modality, *S*_*t*,*t*_^*B*^ for the text modality, and *S*_*v*,*t*_^*B*^ for the cross-modality of image-text between image modality and text modality. *s*_*v*,*v*_^*B*^=cos(*b*_*i*_^*v*^, *b*_*j*_^*v*^)=(*b*_*i*_^*v*^(*b*_*j*_^*v*^)^*T*^/‖*b*_*i*_^*v*^‖_2_‖*b*_*j*_^*v*^‖_2_) ∈ [−1, +1]. Similarly, *s*_*t*,*t*_^*B*^=cos(*b*_*i*_^*t*^, *b*_*j*_^*t*^), *s*_*v*,*t*_^*B*^=cos(*b*_*i*_^*v*^, *b*_*j*_^*t*^). We also measure the similarity of pairs of samples in the feature vectors space and define *S*_*v*,*v*_^*F*^ for the image modality, *S*_*t*,*t*_^*F*^ for the text modality, and *S*_*v*,*t*_^*F*^ for the cross-modality of image-text between image modality and text modality. We use the trained features (*F*^*v*^={*f*_*i*_^*v*^}_*i*=1_^*n*^) to construct the image modal, where *s*_*v*,*v*_^*F*^=cos(*f*_*i*_^*v*^, *f*_*j*_^*v*^). Similarly, *s*_*t*,*t*_^*F*^=cos(*f*_*i*_^*t*^, *f*_*j*_^*t*^) and *s*_*v*,*t*_^*F*^=cos(*f*_*i*_^*v*^, *f*_*j*_^*t*^).

#### 3.3.1. Similarity Semantic Alignment

Because of the difference in the features distribution of cross-modal instances, the semantic description corresponding to the binary hash code often deviates from the semantic description of the feature, leading to some deviations in the search results. However, the original neighborhood relationship of different corresponding modalities are retained for the similarity information of hash codes or features. Although the similarity information is calculated in different modalities, we need to measure it in a common space. Therefore, the core of cross-modal retrieval is to solve the measurement and alignment of similarity information between different modalities.

The article "Deep Unsupervised Hashing for Large-Scale Cross-Modal Retrieval Using Knowledge Distillation Model" was retracted in 2023. Reasons: signs of a paper mill; compromised peer review; unreliable results or conclusions.

To solve this problem, we propose to align the similarity information of different modalities. We calculate the similarity matrix using the cosine similarity function cos (). Firstly, in order to align the similarity information of the hash code from the intramodality with the similarity information of the semantic feature, the defined loss function is as follows:

(1) $$\begin{array}{c} L_{\text{intra}}={\sum \left\|S_{v,v}^{B}-\mu S_{v,v}^{F}\right\|}^{2}+{\sum \left\|S_{t,t}^{B}-\mu S_{t,t}^{F}\right\|}^{2}, \end{array}$$

where *μ* is a trade-off parameter to improve the flexibility of our similarity alignment. Secondly, in order to further align similarity information, we not only align semantic information from intramodality, but also align from intermodality. We align the similarity of instance features with the similarity of hash codes between different modalities:

(2) $$\begin{array}{c} L_{\text{inter}}={\sum \left\|S_{v,v}^{B}-\mu S_{v,t}^{F}\right\|}^{2}+{\sum \left\|S_{t,t}^{B}-\mu S_{v,t}^{F}\right\|}^{2}+{\sum \left\|S_{v,t}^{B}-\mu S_{v,t}^{F}\right\|}^{2}, \end{array}$$

where *S*_*v*,*t*_^*F*^(*i*, *j*) represents the similarity between *i* − th and *j* − th instance, which is obtained by a weighted sum of *S*_*v*,*v*_^*F*^ and *S*_*t*,*t*_^*F*^:

(3) $$\begin{array}{c} S_{v,t}^{F}=\alpha S_{v,v}^{F}+\beta S_{t,t}^{F}+\frac{\gamma }{2}\left(\cos\left(S_{v,v}^{F},S_{t,t}^{F}\right)+\cos\;{\left(S_{v,v}^{F},S_{t,t}^{F}\right)}^{T}\right)\text{,}\;\text{s.t. }\alpha ,\beta ,\gamma \geq 0,\alpha +\beta +\gamma =1, \end{array}$$

where *α*, *β*, and *γ* are trade-off parameters, which are used to adjust the similarity relationship of different modalities. Finally, we merge the similarity alignment loss of the intermodality and that of the intramodality:

(4) $$\begin{array}{c} L_{S}=L_{\text{inter}}+L_{\text{intra}}. \end{array}$$

#### 3.3.2. Diagonal Semantic Alignment

Looking closely at the cross-modal similarity matrix, we find that the diagonal elements of the matrix *S*_*v*,*t*_^*B*^ are calculated between the image-text pair hash code, so any diagonal member of the matrix should be equal to 1. In order to minimize the quantization error of diagonal elements and increase the similarity between hash codes of the same label, we can define the following formula:

(5) $$\begin{array}{c} L_{\text{diag}}=\underset{B_{v},B_{t}}{\min}\sum_{i=1}^{n}{\left\|1-S_{v,t}^{B}\left(i,i\right)\right\|}^{2}. \end{array}$$

In addition, the image-text pairs of off-diagonal elements in a matrix are the same as those of its symmetric elements. For example, the symmetric element of *S*_*v*,*t*_^*B*^(1,2) is *S*_*v*,*t*_^*B*^(2,1), both of whose label-pairs consist of the label of the 1st image-text pair and the label of the 2nd image-text pair. Therefore, we can unify off-diagonal elements by minimizing symmetric loss:

(6) $$\begin{array}{c} L_{\text{off}-\text{diag}}=\underset{B_{v},B_{t}}{\min}\frac{1}{2}\overset{n}{\underset{i=1}{\sum }}\overset{n}{\underset{j}{\sum }}{\left\|S_{v,t}^{B}\left(i,j\right)-S_{v,t}^{B}\left(j,i\right)\right\|}^{2}. \end{array}$$

Finally, the diagonal alignment loss is formulated as

(7) $$\begin{array}{c} L_{D}=L_{\text{diag}}+L_{\text{off}-\text{diag}}. \end{array}$$

We combine the similarity alignment loss and diagonal alignment loss in the teacher module to get the final unsupervised teacher model loss, as shown below:

(8) $$\begin{array}{c} \underset{B_{v},B_{t}}{\min}L=L_{S}+L_{D}, \end{array}$$

where *L*_*S*_ and *L*_*D*_ are the similarity alignment loss and the diagonal alignment loss, respectively.

The article "Deep Unsupervised Hashing for Large-Scale Cross-Modal Retrieval Using Knowledge Distillation Model" was retracted in 2023. Reasons: signs of a paper mill; compromised peer review; unreliable results or conclusions.

### 3.4. Supervised Student Model

After unsupervised training of teacher model, we obtained soft similarity matrix *S*^*O*^. In order to maintain the semantic correlation of the different modalities, the learning process of the two modals (image and text) is supervised by the similarity matrix *S*^*O*^. Firstly, a good hash code should have good discriminative ability in intramodal to retain semantic information. On the contrary, effective hash codes in each modality can improve the performance of cross-mode retrieval. Therefore, our objective function includes two types: intramodality similarity preservation (intramodality triplet loss) and intermodal similarity preservation (intermodal pairwise and triplet loss).

Inspired by DTSH [5], we use the triplet label as the supervision information to describe the relative semantic relationship between three data to construct the triplet network and to dig out more semantic information and improve the retrieval accuracy. During triplet sampling, it is not feasible to sample all triples at once due to memory size and computational resource constraints. To overcome this problem, we used mini-batch method for triplet sampling. The triplet form of image mode is constructed as follows: (*v*_*i*_, *t*_*j*_^+^, *t*_*k*_^−^); text instance *t*_*k*_^−^ is semantically unrelated to image *v*_*i*_, while *t*_*j*_^+^ is the opposite. Similarly, the text modality triplet form (*t*_*i*_, *v*_*j*_^+^, *v*_*k*_^−^). In order to better retain the semantic similarity of training samples in hamming space and enhance the discriminability of learned hash codes, the objective function is divided into two parts: (1) the intramodal triplet loss and (2) the intermodal triplet loss.

The article "Deep Unsupervised Hashing for Large-Scale Cross-Modal Retrieval Using Knowledge Distillation Model" was retracted in 2023. Reasons: signs of a paper mill; compromised peer review; unreliable results or conclusions.

#### 3.4.1. Intramodal Triplet Loss

In order to further make the generated hash code more accurate, it is necessary to not only retain the semantic similarity across modalities, but also to mine the essential semantic information in each modal to enhance the discriminability of the hash code, thereby improving the retrieval performance of cross-modal retrieval. Therefore, we introduce the intramodal triplet loss as part of the objective function. The intramodal triplet loss in the image modal can be obtained as follows:

(9) $$\begin{array}{c} L_{\text{tri}-\text{intra}}v=-\log\;p\left(T|H^{v}\right)=-\underset{i,j,k}{\sum }\log\;p\left(\left(v_{i},v_{j}^{+},v_{k}^{-}\right)|H^{v}\right)\\ =-\underset{i,j,k}{\sum }\left(\theta_{v_{i}v_{j}^{+}}-\theta_{v_{i}v_{k}^{-}}-\omega -\log\left(1+e^{\theta_{v_{i}v_{j}^{+}}-\theta_{v_{i}v_{k}^{-}}-\alpha }\right)\right), \end{array}$$

where *θ*_*v*_*i*_*v*_*j*_^+^_=(1/2)(*H*_*∗v*_*i*__^*v*^)^*T*^*H*_*∗v*_*j*_^+^_^*v*^ and *θ*_*v*_*i*_*v*_*k*_^−^_=(1/2)(*H*_*∗v*_*i*__^*v*^)^*T*^*H*_*∗v*_*k*_^−^_^*v*^. Similarly, the intramodal triplet loss in the text modal can be obtained as follows:

(10) $$\begin{array}{c} L_{\text{tri}-\text{intra}}t=-\sum_{i,j,k}\left(\theta_{t_{i}t_{j}^{+}}-\theta_{t_{i}t_{k}^{-}}-\omega -\log\left(1+e^{\theta_{t_{i}t_{j}^{+}}-\theta_{t_{i}t_{k}^{-}}-\alpha }\right)\right)\\ =-\sum_{i,j,k}\left(\theta_{t_{i}t_{j}^{+}}-\theta_{t_{i}t_{k}^{-}}-\omega -\log\left(1+e^{\theta_{t_{i}t_{j}^{+}}-\theta_{t_{i}t_{k}^{-}}-\alpha }\right)\right), \end{array}$$

where *θ*_*t*_*i*_*t*_*j*_^+^_=(1/2)(*H*_*∗t*_*i*__^*t*^)^*T*^*H*_*∗t*_*j*_^+^_^*t*^ and *θ*_*t*_*i*_*t*_*k*_^−^_=(1/2)(*H*_*∗t*_*i*__^*t*^)^*T*^*H*_*∗t*_*k*_^−^_^*t*^. By adding equations (9) and (10), the intramodal triplet loss can be obtained as follows:

(11) $$\begin{array}{c} L_{\text{tri}-\text{intra}}=L_{\text{tri}-\text{intra}}v+L_{\text{tri}-\text{intra}}t. \end{array}$$

#### 3.4.2. Intermodal Triplet Loss

In order to achieve effective cross-modal hashing retrieval, we add the intermodal triplet loss to the objective loss function to effectively capture the heterogeneous correlation cross modal. Therefore, the intermodal triplet loss from image to text is as follows:

(12) $$\begin{array}{c} L_{\text{tri}-\text{inter}}v=-\log\;p\left(T|H^{v},H^{t},H^{t}\right)=-\sum_{i,j,k}\log\;p\left(\left(v_{i},t_{j}^{+},t_{k}^{-}\right)|H^{v},H^{t},H^{t}\right)\\ =-\sum_{i,j,k}\left(\theta_{v_{i}t_{j}^{+}}-\theta_{v_{i}t_{k}^{-}}-\omega -\log\left(1+e^{\theta_{v_{i}t_{j}^{+}}-\theta_{v_{i}t_{k}^{-}}-\alpha }\right)\right), \end{array}$$

where *θ*_*v*_*i*_*t*_*j*_^+^_=(1/2)(*H*_*∗v*_*i*__^*v*^)^*T*^*H*_*∗t*_*j*_^+^_^*t*^ and *θ*_*v*_*i*_*t*_*k*_^−^_=(1/2)(*H*_*∗v*_*i*__^*v*^)^*T*^*H*_*∗t*_*k*_^−^_^*t*^. Similarly, the intermodal triplet loss from text to image is as follows:

(13) $$\begin{array}{c} L_{\text{tri}-\text{inter}}t=-\sum_{i,j,k}\log\;p\left(\left(t_{i},v_{j}^{+},v_{k}^{-}\right)|H^{t},H^{v},H^{v}\right)\\ =-\sum_{i,j,k}\left(\theta_{t_{i}v_{j}^{+}}-\theta_{t_{i}v_{k}^{-}}-\omega -\log\left(1+e^{\theta_{t_{i}v_{j}^{+}}-\theta_{t_{i}v_{k}^{-}}-\alpha }\right)\right), \end{array}$$

where *θ*_*t*_*i*_*v*_*j*_^+^_=(1/2)(*H*_*∗t*_*i*__^*t*^)^*T*^*H*_*∗v*_*j*_^+^_^*v*^ and *θ*_*t*_*i*_*v*_*k*_^−^_=(1/2)(*H*_*∗t*_*i*__^*t*^)^*T*^*H*_*∗v*_*k*_^−^_^*v*^. By adding equations (12) and (13), the intermodal triplet loss can be obtained as follows:

(14) $$\begin{array}{c} L_{\text{tri}-\text{inter}}=L_{\text{tri}-\text{inter}}v+L_{\text{tri}-\text{inter}}t. \end{array}$$

Obviously, the optimization of formula (14) can reduce the hamming distance between the anchor sample and the positive sample while increasing the hamming distance between the anchor sample and the negative sample, so as to retain as much higher-order semantic information of the sample as possible. By adding the intermodal triplet loss and the intramodal triplet loss, the total triplet loss can be obtained as follows:

(15) $$\begin{array}{c} L_{\text{triplet}}=L_{\text{tri}-\text{inter}}+L_{\text{tri}-\text{intra}}. \end{array}$$

The article "Deep Unsupervised Hashing for Large-Scale Cross-Modal Retrieval Using Knowledge Distillation Model" was retracted in 2023. Reasons: signs of a paper mill; compromised peer review; unreliable results or conclusions.

#### 3.4.3. Intermodal Pairwise Loss

The hash codes from different modalities can effectively preserve semantic similarity. It is a very natural choice to use intermodal pairwise loss in cross-modal retrieval. The intermodal likelihood of pairwise labels is expressed as

(16) $$\begin{array}{c} p\left(S_{ij}|H_{*i}^{v},H_{*j}^{t}\right)=\left\{\begin{array}{c} \sigma \left(\Omega_{ij}^{v,t}\right),s_{ij}=1,\\ 1-\sigma \left(\Omega_{ij}^{v,t}\right),s_{ij}=0. \end{array}\right. \end{array}$$

where Ω_*ij*_^*v*,*t*^=(1/2)*H*_*∗i*_^*v*^*H*_*∗j*_^*t*^ and *σ*(Ω_*ij*_^*v*,*t*^)=(1/(1+*e*^−Ω_*ij*_^*v*,*t*^^)); hash codes of text modality output from TextNet_S are *H*_*∗i*_^*v*^=*f*^*v*^(*v*_*i*_, *θ*_*v*_) and *H*_*∗j*_^*t*^=*f*^*t*^(*t*_*j*_, *θ*_*t*_). Therefore, the intermodal pairwise loss is expressed as

(17) $$\begin{array}{c} L_{\text{pairwise}}=-\log\;p\left(S^{o}|H^{v},H^{t}\right)\\ =-\sum_{s_{ij}^{o}\in S^{o}}\left(s_{ij}^{o}\Omega_{ij}^{v,t}-\log\left(1+e^{\Omega_{ij}^{v,t}}\right)\right). \end{array}$$

Optimization formula (17) can reduce the hamming distance between two similar instances with different modalities and expand the hamming distance between two different instances. Thus, semantic similarity between different modalities instances can be preserved. The overall objective function is written as below:

(18) $$\begin{array}{c} L_{\text{student}}=L_{\text{pairwise}}+L_{\text{triplet}}+\lambda \left({\left\|B-H^{v}\right\|}_{F}^{2}+{\left\|B-H^{t}\right\|}_{F}^{2}\right)\\ \text{s.t. }B\in {\left\{-1,+1\right\}}^{k\times n}, \end{array}$$

where ‖*B* − *H*^*v*^‖_*F*_^2^ and ‖*B* − *H*^*t*^‖_*F*_^2^ are the regularization terms and *λ* are trade-off parameters.

The article "Deep Unsupervised Hashing for Large-Scale Cross-Modal Retrieval Using Knowledge Distillation Model" was retracted in 2023. Reasons: signs of a paper mill; compromised peer review; unreliable results or conclusions.

### 3.5. Models and Implementation Details

For the unsupervised teacher model, suggested by [28–30], we use the VGG19 [35] network as the backbone network to extract image feature, and the last classification layer fc8 is replaced by a hashing layer. In particular, we extract the 4,096-dimensional vectors from the fc7 layer after ReLU activation as the original image features. Meanwhile, for the text modality, we use BoW to embed textual features. TextNet_T consists of two fully connected layers and generates continuous features.

On the other hand, for the supervised student model, inspired by SSAH [15], we use part of its network structure, retaining the image network and the text network, but discarding its discriminative module. The model consists of two deep neural networks, which are used for image modality and text modality, respectively. The batch size of ImageNet_S and TextNet_S is fixed at 128. The dimension of the feature space of the two networks is 4096, and the dimension of the hash space is the same as the length of the hash code. We analyze the hyperparameters sensitivity as reported in Figure 3. In addition, the deep learning framework used in the experiment was TensorFlow V1.15, and the deep learning acceleration card was NVIDIA GTX 1070TI GPU.

## 4. Experiment

We conducted adequate experiments on two popular benchmark datasets NUS-WIDE [36] and MIRFLICKR-25K [37] to prove its performance.

### 4.1. Datasets

MIRFLICKR-25K contains 25015 images, each of which has a corresponding text description, so each instance sample is an image-text pair. There are 24 categories in this dataset, and each instance sample is marked by at least one tag. We used 20,015 samples, of which 2,000 were used as query sets and the rest were used for retrieval. We extracted a 4096-dimensional feature vector from the pretrained 19-layer VGGNet to represent each image and represented each text sample as a 1386-dimensional BoW vector.

NUS-WIDE dataset is a relatively large dataset with 269,498 images and 81 labels. Each image corresponds to some text description. We kept the 10 most common concepts, so we ended up with 186,577 text-image pairs. We retain 1% (1865) of the data as a query database and the rest as a retrieval set. Each image is represented by 4096-dimensional feature vector, and each text is represented by 1000-dimensional BoW vector. In our experiment, the specific implementation details of the two cross-modal datasets are shown in Table 1.

The article "Deep Unsupervised Hashing for Large-Scale Cross-Modal Retrieval Using Knowledge Distillation Model" was retracted in 2023. Reasons: signs of a paper mill; compromised peer review; unreliable results or conclusions.

### 4.2. Evaluation Metric

In order to verify the feasibility of our method, we use two evaluation criteria to evaluate the proposed method: mean average precision (MAP) and top-*K* precision curve. MAP is one of the most commonly used indicators to jointly evaluate search accuracy and ranking. The top-*K* precision represents the accuracy under different numbers of retrieval instances. In the experiment, we use two retrieval tasks for cross-modal retrieval: image-query-text (to retrieve text through image query) and text-query-image (to retrieve image through text query).

### 4.3. Experiment Results

We have selected some representative methods for comparison to verify the effectiveness of the proposed SAKDH method. There are a total of 8 unsupervised hashing methods, including four shallow cross-modal hashing methods and four deep cross-modal hashing methods. CVH [7], IMH [11], CMFH [24], and LSSH [26] are shallow methods, while DBRC [31], UDCMH [28], DJSRH [29], and JDSH [27] are deep methods. For fairness, the comparison method applies the same settings as in the original work.

#### 4.3.1. Results on MIRFLICKR

Table 2 shows the results of MAP@50 on MIRFLICKR, including two cross-mode retrieval tasks with four different length hash codes. The top-*K* precision curves are shown in Figures 3(a) and 3(b). It can be seen from the table that compared to all comparison methods, SAKDH is always the best. In particular, compared to the best unsupervised shallow method CMFH, our method improved by more than 23.3% and 19.5% for different hash code lengths in two retrieval tasks on MIRFLICKR. Compared to the previous best model (JDSH), our method still gets the best results; we achieve improvements of 2.2%, 2.3%, 1.1%, and 1.3% in image-to-text retrieval tasks for different bits, respectively. We plotted the top-*K* precision curves for all the methods. We observed that SAKDH maintained optimal performance throughout for both the image-to-text task and text-to-image tasks. This suggests that our approach improves accuracy through semantic alignment and knowledge distillation.

#### 4.3.2. Results on NUS-WIDE

Table 3 lists the MAP@50 results of all methods on NUS-WIDE. We further plotted the top-*K* precision curves in Figures 3(c) and 3(d). NUS-WIDE is a difficult and challenging dataset. Compared with MIRFLICKR, which has more samples and more complex contents, our approach still leads, but by a smaller margin than MIRFLICKR. Compared with JDSH, our approach still holds the lead. It is important to note that only SAKDH can distill and retain the similarity of different instances, resulting in better performance than other methods. In addition, SAKDH can further improve performance by distilling some data pairs to learn more accurate similarity relationships. From Figure 3, the accuracy of our method remains relatively stable, unlike other methods, when the number of retrieval points is large, the accuracy decreases obviously.

The article "Deep Unsupervised Hashing for Large-Scale Cross-Modal Retrieval Using Knowledge Distillation Model" was retracted in 2023. Reasons: signs of a paper mill; compromised peer review; unreliable results or conclusions.

The above experimental results on these two datasets verify the superiority of SAKDH and indicate that our method can confirm its effectiveness for cross-modal retrieval and bridge modality gap better than other comparison methods.

### 4.4. Ablation Study

In order to further prove the effectiveness of each part of SAKDH, we designed several variants to evaluate the impact of different modules and prove the superiority of SAKDH. The three variants are listed as follows:

1. SAKDH-1 is the variant without diagonal alignment module.
2. SAKDH-2 is the variant without similarity alignment module.
3. SAKDH-3 is the variant without the student module.

We take the MIRFLICKR-25K dataset as an example to show the results of each module, as shown in Table 4. It can be seen that each module plays a certain role in SAKDH. Specifically, the results of SAKDH-1 show that the diagonal alignment module can reduce errors and deviations caused by the asymmetry between the similarity matrices of I2T and T2I. The results of SAKDH-2 indicate the importance of the similarity alignment module, which can align hash codes and features from different modalities. Besides, the performance of SAKDH-3 shows that the student module will significantly improve the MAP results, so the student module is a very important component.

### 4.5. Parameter Sensitivity

In deep learning, the adjustment of hyperparameters may have a very important impact on the system. In this section, we evaluated the impact of several trade-off parameters on the results. Taking the results of MAP@50 on MIRFLICKR as an example, Figures 4(a)–4(c) show the results of precision@top-*K*. The parameter *μ* can greatly improve the flexibility of our similarity alignment. We adjusted the parameter *μ* and got the best results at *μ*=2.5. At the same time, we also observed the impact of parameters *α*, *β*, and *γ* on performance. These three parameters adjust the importance of neighborhood relations in different ways. We cross-validated the hyperparameters *α*, *β*, and *γ* and experimented with the degree of weighing the parameters from 0 to 1. Finally, set *α*=0.5, *β*=0.1, and *γ*=0.4 for MIRFLICKR and set *α*=0.4, *β*=0.3, and *γ*=0.3 for NUS-WIDE.

The article "Deep Unsupervised Hashing for Large-Scale Cross-Modal Retrieval Using Knowledge Distillation Model" was retracted in 2023. Reasons: signs of a paper mill; compromised peer review; unreliable results or conclusions.

## 5. Conclusions

This work presented a novel unsupervised semantic alignment cross-modal hashing method based on knowledge distillation (SAKDH), which can learn a distilled confidence similarity signals. The method guides the supervised method by the distillation information obtained from the unsupervised method. Under the supervision of teacher model distillation information, student model can generate more discriminative hash codes. Compared with several typical unsupervised cross-modal retrieval methods, SAKDH achieves better retrieval performance on two widely used cross-modal datasets.

## Figures and Tables

**Figure 1:** The proposed SAKDH framework consists of two modules: unsupervised teacher model (a) and supervised student model (b). The teacher model is trained in an unsupervised way. By distilling the knowledge from the teacher model, the similarity matrix *S*_*v*,*t*_^*O*^ (soft similarity) is established, and it is used to supervise the student model. The teacher model adopted an unsupervised semantic alignment hashing method, and the student model adopts the joint loss of pairwise and triplet; these loss functions apply not only to intermodal, but also to intramodal.

**Figure 2:** Examples of soft similarity and hard similarity.

**Figure 3:** Precision@top-*K* curves on MIRFLICKR and NUS-WIDE with 128-bit code length. (a) Image-to-text. (b) Text-to-image. (c) Image-to-text. (d) Text-to-image.

**Figure 4:** Parameters' sensitivity analysis on MIRFLICKR. (a) The parameter *μ*. (b) The parameter *α*. (c) The parameter *β*.

**Table 1:** Setup of the two cross-modal datasets.

Dataset	Total	Training set	Test set	Labels	Image feature	Text feature
MIRFLICKR-25k	20,015	18,015	2,000	24	4,096d VGGNet	1,386d BoW
NUS-WIDE	186,577	15,000	1865	10	4,096d VGGNet	1,000d BoW

**Table 2:** The MAP@50 results of two retrieval tasks on MIRFLICKR with various code lengths.

Methods	Image-query-text				Text-query-image			
	16	32	64	128	16	32	64	128
CVH [7]	0.606	0.599	0.596	0.598	0.591	0.583	0.576	0.576
IMH [11]	0.612	0.601	0.592	0.579	0.603	0.595	0.589	0.580
CMFH [24]	0.621	0.624	0.625	0.627	0.642	0.662	0.676	0.685
LSSH [26]	0.584	0.599	0.602	0.614	0.618	0.626	0.626	0.628
DBRC [31]	0.617	0.619	0.620	0.621	0.618	0.626	0.626	0.628
UDCMH [28]	0.689	0.698	0.714	0.717	0.692	0.704	0.718	0.733
DJSRH [29]	0.810	0.843	0.862	0.876	0.786	0.822	0.835	0.847
JDSH [27]	0.832	0.853	0.882	0.892	0.825	0.864	0.878	0.880
Ours	**0.854**	**0.876**	**0.893**	**0.905**	**0.837**	**0.867**	**0.882**	**0.884**

The article "Deep Unsupervised Hashing for Large-Scale Cross-Modal Retrieval Using Knowledge Distillation Model" was retracted in 2023. Reasons: signs of a paper mill; compromised peer review; unreliable results or conclusions.

**Table 3:** The MAP@50 results of two retrieval tasks on NUS-WIDE with various code lengths.

Methods	Image-query-text				Text-query-image			
	16	32	64	128	16	32	64	128
CVH [7]	0.372	0.362	0.406	0.390	0.401	0.384	0.442	0.432
IMH [11]	0.470	0.473	0.476	0.459	0.478	0.483	0.472	0.462
CMFH [24]	0.455	0.459	0.465	0.467	0.529	0.577	0.614	0.645
LSSH [26]	0.481	0.489	0.507	0.507	0.455	0.459	0.416	0.473
DBRC [31]	0.424	0.459	0.447	0.447	0.455	0.459	0.416	0.473
UDCMH [28]	0.511	0.519	0.524	0.558	0.637	0.653	0.695	0.716
DJSRH [29]	0.724	0.773	0.798	0.817	0.712	0.744	0.771	0.789
JDSH [27]	0.736	0.793	0.832	0.835	0.721	0.785	0.794	0.804
Ours	**0.764**	**0.809**	**0.837**	**0.836**	**0.759**	**0.796**	**0.808**	**0.819**

**Table 4:** The MAP@50 results at 128 bits for ablation analysis on MIRFLICKR.

Method	Configuration	I2T	T2I
SAKDH	Teacher (*L*_*S*_+*L*_*D*_) + student	0.905	0.884
SAKDH-1	Teacher (*L*_*S*_) + student	0.893	0.879
SAKDH-2	Teacher (*L*_*D*_) + student	0.876	0.861
SAKDH-3	Teacher (*L*_*S*_+*L*_*D*_)	0.851	0.842

## Data Availability

The datasets supporting this paper are from previously reported studies and datasets, which have been cited. The processed data are available . MIRFlickr can be accessed at http://press.liacs.nl/mirflickr/, and NUS-WIDE at https://lms.comp.nus.edu.sg/wp-content/uploads/2019/research/uswide/NUS-WIDE.html.
